# In Vitro Evaluation of Extracellular Enzyme Activity and Its Biocontrol Efficacy of Bacterial Isolates from Pepper Plants for the Management of *Phytophthora capsici*

**DOI:** 10.1155/2022/6778352

**Published:** 2022-09-26

**Authors:** Mesele Admassie, Yitbarek Woldehawariat, Tesfaye Alemu

**Affiliations:** ^1^Department of Microbial, Cellular and Molecular Biology), Addis Ababa University, Addis Ababa, Ethiopia; ^2^Department of Zoological Science, Addis Ababa University, Addis Ababa, Ethiopia

## Abstract

*Phytophthora capsici* is one of the most devastating fungal pathogens, causing severe diseases that lead to economic loss in the pepper industry. As a result of the infections, the chemical approach is becoming more popular. Biological control, on the other hand, is better suited to controlling fungal pathogens. The biological control approach significantly reduces the problems associated with chemical applications while restoring natural environmental balance. As a result, the overall findings indicate that certain bacterial isolates play a beneficial role in lytic enzyme production and biocontrol activities against *P. capsici*. Bacterial isolates obtained from the pepper plants were screened for lytic enzyme and anti-oomycete activity against *Phytophthora capsici* in Ethiopia. Sixty bacterial isolates were isolated and tested against *Phytophthora capsici*. From these bacterial isolates, different inhibition zones and hydrolytic enzyme production were detected. Biochemical tests using an automated machine (MALDI-TOF, VITEK 2 compact and 16S rRNA) revealed that three of them, AAUSR23, AAULE41, and AAULE51, showed a high inhibition zone and high production of hydrolytic enzymes and were identified as *Enterobacter cloacae* (AAUSR23), *Pseudomonas fluorescens* (AAULE41), and undetermined (AAULE51). The effects of diffusable metabolite isolate AAULE51 has a 66.7% inhibition zone against *Phytophthora capsici*, followed by AAULE41 and AAUSR23, which have 59.7% and 14.1% inhibition zones, respectively. These bacterial isolates showed high production of hydrolytic enzymes like protease, cellulase, chitinase, and lipase (5-34 diameter of inhibition zone). As a result, the overall findings show that selected bacterial isolates play a beneficial role in lytic enzyme production and for their biocontrol activities against *P. capsici*.

## 1. Introduction

A soil-borne disease is the most likely cause of continuous cropping obstacles in pepper plants. Increasing the production of agriculture is a global necessity to feed the accelerating population with limited cultivable agricultural land. To achieve this goal, synthetic fertilizers and pesticides have been used indefinitely, causing environmental damage. Substituting these synthetic chemicals with biocontrol agents is an environmentally friendly alternative [1].

Antagonistic bacterial isolates show biocontrol ability in soil-borne disease management [2, 3]. Fungal endophytes with a broad spectrum of pathogen control spectrum and host adaptability reduce biotic stress in agriculturally important crops [4]. In addition to the production of antibiotics, antagonistic bacterial isolate*s* also produce extracellular enzymes [5]. Extracellular enzymes produced by various microorganisms are used as hydrolytic enzymes, degrading the cell wall structural components of most fungi [6, 7]. Extracellular enzymes are required for the degradation of the fungal pathogen mycelia [8]. Plant diseases have been managed with microbial lytic enzymes such as chitinase and b-1,3-glucanase. Chitin is an insoluble polysaccharide found in the cell walls of fungi, insect gut walls, and worms, which can be hydrolyzed by bacteria [8]. Bacterial hydrolytic enzymes (e. g., cellulase, chitinase, catalase, and proteases) have been studied until now in the infection process and pathogenesis of plants [9]. Varieties of hydrolytic enzymes produced by the rhizosphere's microbial community are responsible for the breakdown of different components of fungal pathogens [10]. Previous studies [11, 12] have mostly focused on the induction of extracellular enzymes produced by fungus and bacteria. Therefore, alternative control techniques for the control of *Phytophthora* blight disease should be developed. Biological control is regarded as an effective, safe, and environmentally friendly method of managing plant diseases. In several crops, *Pseudomonas* spp. has been widely used as a biological control agent against a wide range of soil-borne diseases [13]. The rhizosphere bacteria, in addition to the antagonistic effect of plant pathogens, are also used as crop-enhancers and biofertilizers [14]. The combination of leaf extract with plant growth-promoting bacteria inhibited plant pathogens and increased its yield and quality [15]. Lytic enzymes are among the mechanisms used by *Pseudomonas* spp. to suppress diseases [16]. Jadhav et al. [17] investigated the production of proteases from rhizosphere bacteria and their application for the biocontrol of plant pathogens, which has not been thoroughly investigated and requires further research for the development of an efficient bioprocess.

This study is aimed at examining bacterial isolates obtained from various parts of pepper plants in Southeastern Ethiopia, in terms of their activity to produce lytic enzymes like proteases, cellulases, chitinases, lecithinase, and lipases, as well as to evaluate their anti-oomycete effect against *P. capsici*.

## 2. Methods and Materials

### 2.1. Sample Collection

Two hundred bacterial isolates were collected from the rhizosphere and tissues of pepper plants from two locations: Adama (8.54°N, 39.27°E) and Ziway (7°55' N, 8° 43' 0.01” E), across Southeastern Ethiopia.

### 2.2. Isolation of Bacterial and Fungal Antagonists

Samples of rhizosphere soil were collected from all farms surveyed by pulling up the healthy pepper plants carefully without injuring their root systems. It is then gently shacked to remove any excess soil before being sent to the laboratory in a sterile polythene bag. Fungal and bacterial spp. were isolated using the recommended medium. The procedure was carried out as follows.

To obtain a 1 : 10 (10^−1^) dilution, ten grams of soil samples were obtained separately, suspended in 90 ml of sterile distilled water, and shaken at 180 rpm. To make 1 : 100 (10^−2^) dilutions, one ml of this was transferred to a test tube with nine ml of sterile distilled water. To get a 1 : 1000(10^−3^) dilution, one ml of this was transferred to a test tube containing nine ml of sterile distilled water. Similarly, 10^−4^ dilution was used for fungal spp. isolation while 10^−5^ dilution was used for bacterial spp. isolation. One hundred microliters of each dilution were pipped into Petri plates, containing 20 ml of separate sterile and cooling media, and each treatment was replicated three times. Representative fungal and bacterial colonies were selected, purified, and stored at −20°C for future use.

#### 2.2.1. Isolation of Endophyte Bacteria

Five grams of leaf, stem, and root were collected separately to represent the samples from the whole plant. Endophytic bacterial isolates were obtained from the leaves, stems, and roots of each pepper plant following the methods [18]. The plant parts were surface sterilized and ground separately with a waring blender. Endophytic bacteria were isolated from the internal tissues of roots and stems of healthy looking pepper plants collected from the Southeastern parts of Ethiopia's pepper growing regions such as “Meki” and “Wonji” districts. Surface sterilization was performed for one minute with 1% sodium hypochlorite and 70% alcohol, followed by rinsing five times in sterile distilled water. Surface sterility was checked for each sample to regulate the effect of the disinfection procedure. For this, 0.1 ml of the last wash was transferred to 9 ml of NAB incubated at 28°C and spread onto NA plate for a sterility check. The tissue samples (5.0 g) were ground in phosphate-buffered saline (PBS) aseptically and centrifuged (60 g) for a minute. The supernatant was serially diluted up to 10^5^ before being poured onto NA plates. They were incubated at 28°C for 72 hours, purified, and maintained on skim milk, tryptone, glucose, and glycerin (STGG).

#### 2.2.2. Isolation of *P. capsici*

Isolation of *P. capsici* was conducted according to the method of Zheng (1997). Infected peppers which showed a *P. capsici* symptoms were collected from diseased fields in Southeastern Ethiopia. After being rinsed with tap water, the tissues between the infected and healthy parts of peppers were cut into two to three pieces and then plated on a rose bengal agar medium (papaic digest of soybean meal 5 g, dextrose 10 g, monopotassium phosphate 1 g, magnesium sulfate 0.5 g, rose bengal 0.05 g, and agar 20 g/l) for *P. capsici*. Following inoculation for 5 days at 28°C, the isolates were purified by picking out the mycelia at the edge of the colony and transferring them to PDA medium, followed by incubating for five days under the same conditions. After purification, mycelial plugs were cut with a scalpel and inoculated back to pepper plants, and the isolates that caused symptoms similar to those of plants in fields were used for the identification of the pathogen.

#### 2.2.3. Identification of *P. capsici.*

For identification of *P. capsici*, the purified isolates were transferred to the center of Petri plates of PDA medium and cultivated at 28°C for five days, the refreshed *P. capsici* identified using MALD-TOF semi-automated machine following [19].

### 2.3. Maintenance of Pure Culture

#### 2.3.1. Maintenance of the Fungal Pure Culture

The fungus was subcultured on PDA slants and incubated at 28°C for 14 days. Such slants were preserved in refrigerator at −20°C and maintained. Subculturing was done once a month. Such cultures were used throughout the study.

#### 2.3.2. Maintenance of the Bacterial Pure Culture

The bacteria were subcultured in nutrient and 5% sheep blood base agar plates for 72 hours before being stored in skim milk, tryptone, glucose, and glycerin (STGG) at −20°C and maintained.

### 2.4. Identification

#### 2.4.1. Bacterial Identification

*(1) Identification of Bacterial Isolates Using MALDI-TOF MS*. For bacterial identification using the MALDI-TOF MS method, a single pure colony was taken from the nutrient agar of each isolate with the help of a sterile toothpick and placed onto a special steel 96 micro scout plate (MSP) (Bruker Daltonics) (the direct transfer method). This was spread onto the wells in the plate in the form of a thin film. After drying, one microliter of *α-*cyano*-*4*-*hydroxycinnamic acid (1 *μ*l CHCA) matrix solution (12.5 mg/ml CHCA in a 50% Acetonitrile (CAN) and 2.5% trifluoroacetic acid (TFA) mixture was added and allowed to dry completely at room temperature. The MALDI 96 MSP was placed in the MALDI-TOF MS device, and the system was operated using the optimized method for the identification of microorganisms in linear positive ion mode at a 2,000-20,000 Dalton (Da) mass range. A 60 Hz nitrogen laser was employed at 337 nm as the ion source. To obtain the spectra, laser pulses consisting of 40 packets of 240 were applied in the measurement of each colony [20]. Each sample was studied in triplicate.

*(2) Identification of Selected Bacterial Isolates Using VITEK 2 Compact*. GP ID REF21342 (Identification-Gram-positive bacteria) and GN ID REF21341 (Identification-Gram-negative bacteria) cards are used in the VITEK 2 compact (bioMérieux) system. The VITEK 2 compact is an automated microbiology system utilizing growth-based technology. A sterile swab sample was used to transfer a pure culture and to suspend them in 3 ml of normal saline (NaCl 0.45%, pH 5-7). Then, turbidity was adjusted by DensiCheck to match 0.5–0.6 McFarland, which is the proper inoculum density for Gram-negative and Gram-positive bacteria as stated by the manufacturer.

*(3) Phylogenetic Analysis Based on 16S rRNA Gene Sequencing*. Identification of bacterial isolates using 16S rRNA genes gives a taxonomic status in any bacterial community [21]. Extracted DNA was used to amplify the universal 16S rRNA gene using the following primers: 63f (5′-CAG GCC TAA CAC ATG CAA GTC-3′) and 1387r (5′-GGG CGG WGT GTA CAA GGC-3′). PCR amplification was carried out with the Maxime PCR PreMix Kit and a PCR thermocycler (USA). The PCR reaction mixtures contained 2.5 U of i-Taq™ DNA polymerase (5 U/*μ*l), 2.5 mM of each deoxynucleoside triphosphates (dNTPs), 1X of PCR reaction buffer (10X), 1X of gel loading buffer, and 1 *μ*l of DNA template. The temperature cycle for the PCR was carried out using a method described previously [22]. Sequences were aligned using the BLAST platform (http://www.Ncbi.nlm.nih.gov/BLAST). Phylogenetic analysis of the isolates' sequences with their closest relatives received from GenBank was also used to identify their exact phylogenetic position. Phylogenetic trees were generated using the Maximum Likelihood (ML) technique after the obtained sequences were aligned by multiple sequence alignments using ClusterWand [23]. MEGA 7 with Kimura 2-parameter evolutionary distances were computed [24]. Bootstrap resampling support of the data sets with 1000 replications was used.

### 2.5. Bacterial Isolates and Their Antimicrobial Activity

To test their antibacterial activity, the bacterial isolates were cultured in a nutrient broth medium for 10 days at 28°C on a shaker at 180 rpm. The crude fermentation broth was well mixed and centrifuged at 4000 rpm for 5 minutes. The supernatants were extracted twice with an equal volume of ethyl acetate and shaken vigorously for 20 minutes. The organic solvent extract was then evaporated under reduced pressure using a rotary evaporator (Buchi 461-water bath (6 l), Switzerland) at 40°C to get a crude extract. After being dissolved in ethyl acetate, the crude extracts were tested for antimicrobial screening using the agar diffusion method [25]. Nutrient broth media dissolved in ethyl acetate was used as a control.

After striking with the suspension of a tested organism, the media were cut using a sterile cork borer and filled with 20 *μ*l of bacterial crude extract. Negative control wells were filled with 20 *μ*l of ethyl acetate and the positive controls were filled with 20 *μ*l of 64% mancozeb. The plates were kept in a 4°C refrigerator for 4 hours to allow antimicrobial compounds to defuse before being incubated at 28°C for 72 h [26]. According to the following formula, the inhibitory activity of each concentration was expressed as a percent growth inhibition when compared to the control (solvent only used in the wells):

(1) $$\begin{array}{c} \text{Growth inhibition }\left(\%\right)=\frac{C-T}{C}\times 100, \end{array}$$

where *C* is the diameter of control and *T* is the diameter of the fungal colony with treatment [27]. Each concentration was replicated three times and three separate tests were performed.

#### 2.5.1. Spore Germination Test (Inhibition Zone Test)

*Phytophthora capsici* spores from a 5-day-old potato dextrose broth (PDB) culture were spread over the other 50% potato dextrose agar (PDA) and 50% nutrient agar plates by swabbing and then allowed to dry at 25°C for 30 min. The bacteria isolates were subcultured and allowed to grow for 72 hours in nutrient broths. In a, double layers of sterile filter paper discs (6 mm in diameter) were inoculated with 20 *μ*l of bacterial culture. After being air-dried for 30 minutes, the discs were put onto the 50 percent PDA plus 50 percent NA plates. Controls were discs loaded with 20 *μ*l of uninoculated nutrient broth (NB). After 48 hours of incubation at 28°C, the radius of the clearing zones around the discs were measured [28].

#### 2.5.2. Evaluation of the Effect of Bacterial Isolates against *Phytophthora capsici* via the Production of Volatile Compounds

The inhibition of *P. capsici* growth through the production of volatile compounds was tested using selected potential bacterial isolates in the divided plate method. One-half of the Petri plates split into two compartments were used; one half was filled with NA (bacterial isolates) and the other half was filled with PDA medium (*P. capsici*) [29]. 20 *μ*l of overnight bacterial culture adjusted to an optical density of 600 nm (0.5) was spotted on one half of the divided Petri dish (NA for control plates), while the targets (a plug of mycelium, *P. capsici*) were inoculated on the other half. Plates were sealed with Parafilm and incubated for 5 days at 28°C in the dark before being photographed and measured. The image was analyzed using the digital imaging software ImageJ (http://imagej.nih.gov/ij/). ImageJ's freehand area measurement tool was used to calculate the mycelium area/diameter. Growth was calculated by subtracting the original mycelial surface from the one obtained after the incubation period. This growth value was then computed on the control plates (inoculated only with NA), and its percentage was calculated as mentioned in 2.5. These assays were performed with 3 replicates.

#### 2.5.3. Screening of Bacterial Isolates for Hydrolytic Enzyme Production

The hydrolytic enzyme production of the selected isolates, such as chitinase, cellulase, protease, lipase, and lecithinase, was screened.

*(1) Qualitative Screening of Proteolytic Activity*. All bacterial isolates were tested for proteolytic activity on skim milk agar plates [30]. Twenty microliters of the 72-hour-old culture of each bacterial isolate was added to skim milk agar containing skim milk powder (10%) and agar (2%) to isolate the producer strain. These plates were incubated for 48 h at 28°C and observed for clear zone production around the colony. The clear zones of the proteolytic activity of bacteria around the colony were measured and recorded in mm.

*(2) Qualitative Screening of Cellulolytic Activity*. The cellulolytic experiment was carried out in triplicate by inoculating the isolates into minimal media (MM) supplemented with 0.1% carboxymethyl cellulose (w/v, 0.1 percent NaNO_3_, 0.05 percent MgSO_4_, 0.1% K_2_HPO_4_, 0.1 percent KCl, 0.05 percent yeast extract, 1.5 percent Agar) [31]. After incubation for 5 days at 28°C, the CMC agar plates were flooded with Gram's iodine and allowed to stand at room temperature for around 10 minutes before being washed with 1 M NaCl. The ratio of the clear zone diameter to the colony diameter of CMC hydrolysis was measured and recorded [32]. The diameter of the clear zone around the colonies was calculated using the enzymatic index (EI) [32].

(2) $$\begin{array}{c} \text{EI}=\frac{\text{Clear zone diameter }}{\text{ Colony diameter}}. \end{array}$$

*(3) Qualitative Screening of Chitinase Activity*. Chitinolytic bacteria were screened according to the method [33]. The bacterial isolates were inoculated into colloidal chitin agar medium (NH_4_SO_4_, 1 g/l; KH_2_PO_4_, 0.2 g/l; K_2_HPO_4_, 1.6 g/l; NaClCL, 0.1; MgSo_4_ and FeSO_4_, 0.01 g/l; CaCL, 0.02 g/l; and agar, 20 g/l) and incubated for five days at 28°C. Chitinolytic bacteria were screened based on clear zones of hydrolysis produced after five days of incubation. The colony diameter and clear zone diameter were calculated using the Chitinolytic Index formula [34].

(3) $$\begin{array}{c} \text{CI}=\frac{\text{Clear zone diameter}–\text{Colony diameter }}{\text{ Colony diameter}}. \end{array}$$

*(4) Qualitative Screening of Lecithinase Activity*. The lecithinase activity was checked by preparing nutrient agar supplemented with 1% NaCl and 10% (v/v) egg yolk emulsion. The formation of a white precipitate around or beneath the inoculum spot revealed lecithinase formation [35].

*(5) Qualitative Screening of Lipase Activity*. To test the extracellular lipase production, all the bacterial isolates were separately inoculated on NA media supplemented with various lipids (1%, v/v) such as tween 20, tween 80, egg yolk, and tributyrin. The pH of the media was maintained at 7, and incubation was carried out at 28°C for up to 5 days. Bacterial isolates showed an opaque zone around colonies and were evaluated as lipase positive [36].

### 2.6. Test for Antibiotic Susceptibility

The disk diffusion method on the Hilton agar medium was used to determine antibiotic susceptibility, as specified by the standard criteria [37]. The antibiotics used for susceptibility of selected bacterial isolates were amoxicillin (AMX; 10 *μ*g), ciprofloxacin (CIP; 5 *μ*g), chloramphenicol (C; 30 *μ*g), gentamycin (GM; 10 *μ*g), cotrimoxazole (SXT; 25 *μ*g), tetracycline (TE; 30 *μ*g), and ceftriaxone (CRX; 30 *μ*g). Antibiotic discs were placed on solid media and incubated for 24 hours at 37°C. The results were interpreted as resistant (R), intermediate resistant (IR), or sensitive (S) to antimicrobial drugs based on the CLSI 2020 guidelines of its inhibition zone size.

### 2.7. Statistical Analysis

GraphPad Prism (version 6) was used for statistical analysis. All tests were performed with three to five replicates for each treatment. The data were tested at least twice with the same results. Treatment groups were evaluated using ANOVA and the test for least significant differences at a probability threshold of 5% (*P* < 0.05).

## 3. Results

### 3.1. Isolation and Identification of Antagonistic Bacteria

Bacteria (200 samples) were isolated from pepper roots, leaves, stems, and rhizosphere. Different biochemical tests were demonstrated to know the antagonistic ability of isolates, AAULE51 and AAULE41, which produced the highest inhibition zones against the mycelial growth of *P. capsici* that were isolated from the leaves of pepper plants. Bacterial isolates, which were used for this experiment, were identified to species level by using the automated MALDI-TOF, VITEK 2 compact machines, and 16S rRNA sequence analysis (Table 1 and Figure 1).

### 3.2. Spore Germination Test (Inhibition Zone Test)

The results of the spore germination test were analyzed by observing the inhibition zones formed by bacterial isolates towards *P. capsici*. The radii of the inhibition zones were measured from the center of the discs to the edge of the inhibition zone. The result was considered positive if an inhibition zone was formed, while the result was negative if the bacteria could not produce inhibition zones.  Figure 2 shows the radius of the inhibition zone obtained in the spore germination test. Isolate AAULE51 had the largest inhibition zone radius of 17.7 mm, while isolate AAULE41 had the smallest radius of 5.1 mm.

### 3.3. Antifungal Activity of Crude Metabolites of Selected Bacterial Isolates

The antimicrobial activity of the bacterial isolates against *Phytophthora capsici* using crude extracts of AAULE41, AAULE51, AAUFE29, and AAUSR23 suppressed the growth of *P. capsici*, respectively. The crude extracts of these isolates showed an inhibitory effect against the *P. capsici*, with a clear zone of 31.5 mm, 16.1 mm, 3.4 mm, and 7.8 mm, respectively, when compared to the control (51.8 mm) (Figure 3 and Table 2).

### 3.4. In Vitro Inhibition of Mycelial Growth of *P. capsici* by Volatile Substances

AAULE41 and AAULE51 isolates produced volatile compounds that inhibited *P.capsici* mycelial growth in vitro. Each significantly reduced mycelial growth, with AAULE41 and AAULE51 having mean mycelial growth of 18.3 mm and 15.1 mm, respectively, compared to 45 mm in the control (Figures 4(a)–4(c)). The isolates' inhibition ability varied significantly (*P* < 0 · 05); AAULE-51 consistently showed the highest inhibition (66·7%) followed by AAULE41 (59.7%) (Figures 4(a) and 4(b)).

### 3.5. Screening for Hydrolytic Enzyme Production Activity

The bacterial isolates that produce various hydrolytic enzymes have an antagonistic effect on the soil fungi. Thus, the bacterial antagonists retrieved in this study were phenotypically characterized in vitro to explore possible mechanisms of antagonistic activity based on protease, cellulase chitinase, lecithinase, and lipase production. The production of at least one type of lytic enzyme (including proteases, lipases, chitinase, lecithinase, and cellulases) was observed in 10–78.3% (10–47/60) of the isolates. The primary type of lytic enzyme produced by bacterial isolates was chitinase, followed by cellulase, and the least common lytic enzyme produced was lichtinase (Figures 5 and 6 and Table 3).

#### 3.5.1. Qualitative Screening of Proteolytic Bacteria

The proteolytic activities of sixty bacterial isolates were assayed using skim milk agar and were demonstrated by the diameter of the clear zone. As shown in Figure 5(a), among the sixty isolates, 23 isolates showed proteolytic activity. Of these, AAUFE13, AAUFE14, AAUFE11, AAUFE10, AAUSR49, and AAULE51 showed high proteolytic activity among the isolated bacteria.

#### 3.5.2. Qualitative Screening of Cellulolytic Activity

In a cellulolytic assay, seventeen of sixty isolates were able to digest cellulose in a medium containing carboxymethyl cellulose. The highest value of the enzymatic index was shown by the AAUSR52 isolate, followed by AAUSR23, AAULE51, AAUSR48, and AAUSR47, with a value index of 9.1, 5.6, 4.4, 2.6, and 2.5, respectively (Figure 5(b)).

#### 3.5.3. Qualitative Screening of Chitinase Activity

The chitinolytic activity was shown by forty-seven out of sixty isolates that formed a clear zone around the colony (Figure 5(c)). The AAUSR42 isolate has the highest chitinolytic index value (1.156) (Figure 2(b)), followed by AAUSR52, AAUSR43, and AAULE51, with a range of 0.258 to 0.534.

#### 3.5.4. Qualitative Screening of Lecithinase Activity

In the present study, detection of various lecithinase activities revealed that among the sixty tested isolates only six isolates had produced lecithinase enzyme (Figure 5(d)).

#### 3.5.5. Qualitative Screening of Lipase Activity

All sixty strains were screened for their potential lipolytic activity, and only 15 of them were shown to have a clear zone around the colonies. The maximum zone of inhibition was shown in three strains, which were named AAUSR1, AAUSR17, and AAUSR58 (Figure 5(e)).

### 3.6. Antibiotic Assay

The selected bacterial isolates showed a distinct zone of inhibition against some antibiotics, i.e., penicillin G, amoxicillin, gentamycin, cotrimoxazole, ciprofloxacin, tetracycline, ceftriaxone, and chloramphenicol. Among bacterial isolates, 100% of isolates were resistant to penicillin G, amoxicillin, and tetracycline; 75% were resistant to cotrimoxazole and ceftriaxone; 50% and 25% were resistant and intermediate to chloroamphenicol, respectively, and 25% were resistant to gentamycin, whereas none of the bacterial isolates were resistant to ciprofloxacin (Table 1).

### 3.7. Molecular Identification of Potential Bacterial Isolates

Phylogenetic trees of three Gram-negative bacterial strains constructed from 16S rRNA sequences showed that the selected isolates were mainly members of the genera *Pseudomonas*, *Rhizobium*, and *Enterobacter* (Figure 1). The sequences of isolates AAUSR23, AAUFE29, and AAULE41 showed 100% similarity. Isolates AAULE41, AAULE29, and AAUSR23 had 100% homology with *Pseudomonas fluorescens, Rhizobium* sp.*, and Enterobacter hormaechei,* respectively (Figure 1).

## 4. Discussions

During crop cultivation, biotic stress resulting from plant pathogens is a serious challenge that causes enormous economic losses. Different agrochemicals are currently being employed to control plant diseases. However, their application is difficult due to public concern regarding dangerous residues, the selection of resistant strains of pathogens, and increased expenses for plant protection. The development of microbe-based control methods could produce effective substitutes for managing crop disease.

The spore germination test revealed the strong inhibition ability against *P. capsici* by isolate AAULE51, with the radii of inhibition of 17.7 mm. The result of the inhibition of the fungus in the spore germination test in this study is higher than that reported by [28, 38], who reported an inhibition zone ranging from 14 to 17 mm and 12.5 to 15 mm, respectively. Despite achieving higher inhibition in the dual culture assay, the bacteria isolates AAUSR23 and AAUFE29 had little or no effect on *P. capsici* spore germination.

Twenty microliters (20 *μ*l) cell-free filtrate of AAULE41 and AAULE51 isolates were extracted using ethyl acetate and showed a high antimicrobial effect against *P. capsici*. In comparison, [39] observed suppression of *P. capsici* by the methanol extract of *Xenorhabdus bovienii*, YL002 was at 16.83 *μ*g ml/1, whereas [40] showed that the ethyl acetate extract of *X. bovienii* SN did not cause suppression of the related pathogen *Phytophthora cactorum* at 50 *μ*g ml/1. Although the difference may be attributed to the use of different bacterial strains, organic solvents, and different culture conditions, it is also understood that the disparity may be attributed to varying assay conditions.

The bacterial plant biostimulants, in addition to plant growth promotion, inhibits the microbial/pathogen growth ensues synergistically through several mechanisms, such as antibiosis, volatile organic compound (VOC) production, extracellular enzymatic lysis, and siderophore-mediated inhibition [41]. The present work aims at addressing this issue by isolating potential bacterial antagonists that can be incorporated into disease management strategies.

In this study, 60 isolates of bacteria were isolated from pepper plants and screened for their ability to produce VOCs with antifungal activity against *P. capsici.* Our findings show that VOC production can play an essential role in the biocontrol activity of *P. capsici.* In our study, volatile metabolites of AAULE51 isolates showed maximum inhibition (66.7%) against the tested pathogen, followed by AAULE41 (59.7%), AAUSR23 (14.1%), and AAUFE29 (12%). Lazazzara et al. [42] studied on *Lysobacter* spp. strains and found VOCs production, like pyrazines and pyrrole, which contribute to the suppression of *P. infestans*. Based on these results, we tested the ability of selected bacterial isolates in the laboratory to produce VOCs, hypothesizing that these VOCs may inhibit the growth of soil-borne plant pathogens.

In this study, three bacterial isolates were found to produce diffusible and volatile organic compounds (VOCs) that inhibited the soil-borne phytopathogenic *P. capsici* by 66.7% in vitro. The inhibition of *P. capsici* mycelial growth observed in this investigation could be due to the physiologically active volatile chemicals.

The production of hydrolytic enzymes by PGPR is an essential mechanism against plant pathogens for sustainable plant disease management. These enzymes break down the cell walls of fungal pathogens, causing cell death [7]. Plant growth-promoting bacteria produce hydrolytic enzymes (chitinase, glucanase, protease, and cellulase) which are responsible for the lysis of phytopathogens through hyperparasitism. Antagonistic activities of fungal endophytes are coupled with the synthesis of lysis defense-related enzymes and compounds such as antimicrobial and antifungal metabolites (*β*-1, 3 glucanases, chitinase, cellulose, protease, hydrolyzing enzymes, fumonisin, and beauvericin) that contribute as a biological control for plant pathogens [4]. Antagonistic properties of hydrolytic enzymes against various phytopathogens play an important role in biocontrol [10, 43]. Different hydrolytic enzymes produced by bacterial strains have an antagonistic effect on soil fungi [44]. Antagonistic activities of fungal endophytes are coupled with the synthesis of bioactive defense-related compounds, which produce b-glucoside-degrading enzymes, like, *β*-1, 3 glucanases, chitinase, cellulose, protease, and hydrolyzing enzymes, that contribute to the control of pathogens [4]. Therefore, the bacterial antagonists screened in this study were phenotypically characterized in vitro to demonstrate possible antagonistic activity mechanisms using protease, cellulase, chitinase, lichetinase, and lipase production. So, from these results, it can be revealed that the production of these enzymes would be the most prominent trait among the antagonists. Four selected potential bacterial isolates that showed antagonistic activities were tested for these activities. All of them showed protease and cellulase activity, but none of them was positive for lipase activity. Chitinase activity was observed only in AAULE51 (Table 3). Jabborova et al. [45] studied endophytic bacterial isolates and discovered that most isolates had positive protease activity, and this was followed by lipase and cellulase activities. From these, four endophytic bacterial isolates (GS4, GS6, GS8, and GS9) had antifungal activity against several fungal strains. In this study, the maximum isolates have positive lipase activity and are followed by chitinase, cellulase, and protease activities.

In this study, 12 protease-producing isolates were screened from endophyte and rhizosphere pepper. Two of these isolates, namely AAULE 41 and AAULE 51, isolated from endophyte pepper, have shown high proteolytic activity. A total of 9 protease positive isolates were obtained from the rhizosphere of various crop plants. Two of these isolates, namely HP_RZ17 and HP_RZ19, produced a copious amount of protease [46]. When introduced as an inoculum, PGPR's resistance to various antibiotics may provide an ecological benefit in terms of survival in the rhizosphere.

The continuous use of antibiotics in animals as well as in agriculture is, in turn, contributing to the increasing problems of antibiotic resistance in bacteria. In an environment with multiple stresses, such as antibiotics, bacterial resistance to both stresses would be more ecologically favorable in terms of survival. With these considerations, the antibiotic resistance among PGPR strains was studied, which differed from antibiotic to antibiotic for all PGPR strains. Antibiotic-resistant microbes will adapt to changing environmental conditions faster through the propagation of R-factors than through mutation and natural selection [47, 48]. Similar investigations on antibiotic resistance by PGPR strains have been reported [49]. In our study, multiple antibiotic resistance was shown by selected isolates (AAULE41 and AAULE51) (Table 1). The presence or absence of resistance mechanisms, as well as the differences in growth conditions and exposure to PGPR stress, may be due to variation in antibiotic resistance.

## 5. Conclusions

In conclusion, *Pseudomonas fluorescens* (AAULE41) and AAULE51 (undetermined) were found to have potent hydrolytic enzyme-producing and antifungal activities. In brief, bacterial isolates' attributes of fungal inhibition enabled them to effectively control *P. capsici* in vitro. Further, these isolates significantly showed a large diameter inhibition zone both in the agar well diffusion and the hydrolytic enzyme test. Therefore, these bacterial isolates can be used as potential bioagents for controlling *P. capsici* and are thus capable of decreasing the excessive use of synthetic fungicides in agriculture.

## Figures and Tables

**Figure 1:** The maximum likelihood tree showed that the three strains AAUSR23, AAUFE29, and AAULE41 were closely related to *Enterobacter hormaechei, Rhizobium sp,* and *Pseudomonas fluorescens*, respectively, and had 100% identity.

**Figure 2:** Radii of inhibition zone in spore germination test.

**Figure 3:** Agar well diffusion test for antifungal activity of crude extracts of selected bacterial isolates against *P. capsici*.

**Figure 4:** (a) The antioomycete effect of volatile compounds produced by the bacterial isolates AAULE41 and AAULE51 against the phytopathogen *P. capsici*. (b) Effect of diffusible compounds produced by selected bacterial isolates on *P. capsici* mycelial growth of AAUSR23, AAUFE29, AAULE41, and AAULE51. (c) Percentage growth inhibition of volatile compounds released by the isolates AAUSR23, AAUFE29, AAULE41, and AAULE51 on *P. capsici.* Represent the mean ± SE values (*n* = 3). Different letters above the bar indicate statistically significant differences compared to the control (Tukey-Kramer's HSD test, *P* < 0.05).

**Figure 5:** In vitro evaluation of different bacterial isolates on Petri dishes with colonies surrounded by zones of extracellular enzymatic activity: (a) protease, (b) cellulase, (c) chitinase, (d) Lichtinase, and (e) Lipase.

**Figure 6:** Shows the percentage of bacterial isolates (out of a total of 60) that produce individual hydrolytic enzymes.

**Table 1:** Antibiotic activity of selected bacterial isolates.

Antibiotics	*Enterobacter hormaechei* (AAUSR23)	*Rhizobium* spp. (AAUFE29)	*Pseudomonas fluorescens* (AAULE41)	AAULE51 (undetermined)	Reference		
					S	IR	R
Penicillin G (10 units)	R (0 mm)	R (0 mm)	R (0 mm)	R (0 mm)	—	—	—
Amoxicillin (10 *μ*g)	R (5 mm)	R (7 mm)	R (0 mm)	R (0 mm)	>17	14-16	<13
Gentamycin(10 *μ*g)	S (18 mm)	S (16 mm)	R (6 mm)	S (15 mm)	>15	13-15	<12
Cotrimoxazole (25 *μ*g)	R (10 mm)	S (17 mm)	R (6 mm)	R (9 mm)	>16	11-15	<10
Ciprofloxin(5 *μ*g)	S (27 mm)	S (30 mm)	S (31 mm)	S (30 mm)	>26	22-25	<21
Ceftriaxone (30 *μ*g)	R (18 mm)	S (25 mm)	R(2 mm)	R(5 mm)	>23	20-22	<19
Chloramphenicol(30 *μ*g)	R (12 mm)	S (20 mm)	R (13 mm)	I (15 mm)	>18	13-17	<12
Tetracycline (30 *μ*g)	R (0 mm)	R (10 mm)	R (0 mm)	R (12 mm)	>15	12-14	<11

∙ S = sensitive, IR = intermediate resistant, and R = resistant.

**Table 2:** Bacterial isolates' antimicrobial activities against *P. capsici.*

Bacterial strain	Diameter clear zone (mm)
	*P. capsici*
C	—
AAUSR23	7.8
AAUFE29	3.4
AAULE41	31.5
AAULE51	16.1

C: controls without bacterial inoculation.

**Table 3:** Extracellular enzymatic activities of different bacterial isolates.

Isolate no		HOST PLANT	Diameters of the clear zone (mm)				
	Strain		Plant tissue	Protease	Cellulase	Chitinase	Lipase
C∗	Distilled H_2_O			0^cd^	0^bc^	0^b^	0^c^
AAUSR1	*Bacillus* spp.	Pepper	Rhizosphere	0^cd^	25.2 + 0.3^ab^	0^b^	29.8 + 3^a^
AAUSR2	*Bacillus thuringiensis*	Pepper	Rhizosphere	0^cd^	25.7 + 0.3^ab^	13.8 + 2^ab^	9.6 + 3^b^
AAUSR5	*Achromobacter denitrificans*	Pepper	Rhizosphere	0^cd^	12.2 + 0.3^bc^	0^b^	0^c^
AAUSR6	*Pseudomonas aeruginosa*	Pepper	Rhizosphere	0^cd^	24.4 + 0.3^a^	0^b^	0^c^
AAUSR7	*Stenotrophomonas maltophilia*	Pepper	Rhizosphere	17.5 + 0.4^bc^	0^bc^	5.7 + 2b	0^c^
AAUSR8	*Comamonas testosteroni*	Pepper	Rhizosphere	0^cd^	0^bc^	13.5 + 2^ab^	0^c^
AAUSR9	*Pseudomonas aeruginosa*	Pepper	Rhizosphere	27 + 0.4^a^	0^bc^	0^b^	0^c^
AAURE10	*Pseudomonas aeruginosa*	Pepper	Root	23.8 + 0.4ab	0^bc^	0^b^	0^c^
AARE 11	*Pantoea cheilomeans*	Pepper	Root	34 + 0.4^a^	0^bc^	0^b^	0^c^
AAURE13	*Pseudomonas aeruginosa*	Pepper	Root	0^cd^	0^bc^	0^b^	0^c^
AAUSE14	*Pseudomonas oryzihabitans*	Pepper	Stem	0^cd^	0^bc^	0^b^	0^c^
AASR15	*Serratia marcescens*	Pepper	Rhizosphere	0^cd^	0^bc^	0^b^	4.1 + 3^c^
AAURE16	*Pseudomonas fluorescens*	Pepper	Root	9.5 + 0.4^bc^	0^bc^	0^b^	14.5 + 3^abc^
AAUFE17	*Enterobacter xiangfangensis*	Pepper	Fruit	0^cd^	18.4 + 0.3^abc^	0^b^	0^c^
AAUSR19	*Pseudomonas stutzeri*	Pepper	Rhizosphere	20.8 + 0.4^ab^	14.9 + 0.3^bc^	16.7 + 2^a^	14.4 + 3^abc^
AAUSR20	*Pseudomonas stutzeri*	Pepper	Rhizosphere	0^cd^	8.5 + 0.3^c^	21.5 + 2 ^a^	12.3 + 3^abc^
AAUSR21	*Pseudomonas stutzeri*	Pepper	Rhizosphere	0^cd^	0^bc^	16.8 + 2^a^	13.2 + 3^abc^
AAUSR22	*Enterobacter asburiae*	Pepper	Rhizosphere	0^cd^	0^bc^	0^b^	12.6 + 3^abc^
AAUSR23	*Enterobacter hormaechei*	Pepper	Rhizosphere	5.13 + 0.4^c^	26.7 + 0.3^a^	0^b^	0^c^
AAUSR25	*Pseudomonas putida*	Pepper	Rhizosphere	0^cd^	0^bc^	0^b^	11 + 3^abc^
AAUSR26	*Pantoea* spp.	Pepper	Rhizosphere	0^cd^	0^bc^	0^b^	18.7 + 3^ab^
AAUSE27	*Pseudomonas aeruginosa*	Pepper	Stem	0^cd^	0^bc^	0^b^	
AAURE30	*Enterobacter hormaechei*	Pepper	Rhizosphere	14.8 + 0.4^bc^	0^bc^	0^b^	11.8 + 3^abc^
AAUSE31	*Enterobacter hormaechei*	Pepper	Stem	0^cd^	0^bc^	14.2 + 2^a^	10 + 3^bc^
AAUSE34	*Enterobacter hormaechei*	Pepper	Stem	0^cd^	0^bc^	0^b^	8.6 + 3bc
AAURE35	*Enterobacter cloacae*	Pepper	Root	0^cd^	0^bc^	0^b^	9.2 + 3^bc^
AAULE41	*Pseudomonas fluorescens*	Pepper	Rhizosphere	26.1 + 0.3^a^	5.6 + 2^c^	0^b^	0^c^
AAUSR42	*Enterobacter cloacae*	Pepper	Rhizosphere	0^cd^	22.6 + 0.3^ab^	19 + 2^a^	0^c^
AAUFE43	*Aeromonas hydrophila/caviae*	Pepper	Rhizosphere	23.8 + 0.4ab	0^bc^	17+ 2^a^	0^c^
AAUSE44	*Rhizobium radiobacter*	Pepper	Rhizosphere	0^cd^	0^bc^	6.6 + 2^b^	0^c^
AAUSR46	*Rhizobium radiobacter*	Pepper	Rhizosphere	0^cd^	0^bc^	14.2 + 2^a^	0^c^
AAUSR47	*Aeromonas hydrophila*	Pepper	Rhizosphere	0^cd^	17.97 + 0.3^ab^	15 + 2^a^	0^c^
AAUSR48	*Enterobacter cloacae*	Pepper	Rhizosphere	0^cd^	19 + 0.3^ab^	0^b^	0^c^
AAUSR49	*Serratia marcescens*	Pepper	Rhizosphere	23.7 + 0.4^ab^	0^bc^	19.1 + 2^a^	0^c^
AAULE51	Undetermined	Pepper	Leaf	33.+0.4^a^	24.8 + 0.3^ab^	22.5 + 2^a^	0c
AAUSR52	*Pseudomonas stutzeri*	Pepper	Rhizosphere	0^cd^	31.5 + 0.3a	18.9 + 2a	0^c^
AAUSR56	*Pseudomonas stutzeri*	Pepper	Rhizosphere	0^cd^	0^bc^	0^b^	0^c^
AAUSR58	Undetermined	Pepper	Rhizosphere	0^cd^	0^bc^		22.7 + 3a
AAUSR59	Undetermined	Pepper	Rhizosphere	0^cd^	0^bc^	0^b^	7.7 + 3^bc^

∗: Control without bacterial inoculation. The identities of the bacterial isolates are available in Table 3. Different letters between lines denote that mean values are significantly different (*P* < 0.05) by Tukey's test, mean + Standard Error (SE) (*n* = 3).

## Data Availability

All data generated or analyzed during this study are included in this published article.

## Abbreviations

ANOVA: Analysis of variance
VOCs: Volatile organic compounds
CLSI: Clinical and laboratory standards institute
mm: Millimeter
*μ*g: Microgram
PGPR: Plant growth promoting rhizosphere
%: Percent
*μ*l: Microliter.
